# Lightweight Image Super-Resolution Based on Re-Parameterization and Self-Calibrated Convolution

**DOI:** 10.1155/2022/8628402

**Published:** 2022-09-26

**Authors:** Sufan Zhang, Xi Chen, Xingwei Huang

**Affiliations:** School of Computer and Communication Engineering, Changsha University of Science and Technology, Changsha 410114, China

## Abstract

Image super-resolution technique can improve image quality by increasing image clarity, bringing a better user experience in real production scenarios. However, existing convolutional neural network methods usually have very deep network layers and a large number of parameters, which causes feature information to be lost as the network deepens, and models with a large numbers of parameters are not suitable for deploying on resource-constrained mobile devices. To address the above problems, we propose a novel lightweight image super-resolution network (RepSCN) based on re-parameterization and self-calibration convolution. Specifically, to reduce the computational cost while capturing more high-frequency details, we designed a re-parameterization distillation block (RepDB) and a self-calibrated distillation block (SCDB). They can improve the reconstruction results by aggregating the local distilled feature information under different receptive fields without introducing extra parameters. On the other hand, the positional information of the image is also crucial for super-resolution reconstruction. Nevertheless, existing lightweight SR methods mainly adopt the channel attention mechanism, which ignores the importance of positional information. Therefore, we introduce a lightweight coordinate attention mechanism (CAM) at the end of RepDB and SCDB to enhance the feature representation at both spatial and channel levels. Numerous experiments have shown that our network has better reconstruction performance with reduced parameters than other classical lightweight super-resolution models.

## 1. Introduction

Image super-resolution (SR) is an important technique used in computer vision tasks for image processing. It is a process that enables image reconstruction by learning a nonlinear mapping between a high-resolution (HR) image and its low-resolution (LR) counterpart. Since SR can increase the resolution while preserving as much as possible the image texture details, it plays a significant role in medical imaging [1], security and surveillance imaging [2], remote sensing images, and preprocessing of some advanced computer vision tasks [3,4]. In general, SR is an ill-posed problem because one LR image may correspond to multiple HR images [5].

Recently, deep learning methods [6–11] have demonstrated great value in computer vision tasks. With the development of convolutional neural networks (CNNs), various CNN-based methods for image super-resolution have emerged and have achieved significant performance breakthroughs. Dong et al. [12] first proposed a network (SRCNN) consisting of three convolutional layers to learn the mapping of LR images to HR images. SRCNN upsamples the input image to a larger size before mapping it, increasing computational difficulty and slower model training. To address this issue, Dong et al. [13] introduced FSRCNN by upsampling the feature maps after the network output, which reduces a significant amount of computation and running time. After this, considering that a limited number of CNN layers cannot fully utilize the feature information of LR images, Kim et al. [14] presented the core idea that deepening and widening the network structure can lead to better performance and proposed a 20-layer network (VDSR). VDSR employs residual learning for the first time in the SR task, effectively speeding up the convergence of the network and avoiding vanishing or exploding gradient problems. EDSR [15] removes the batch normalization (BN) layer, which is disadvantageous to the SR task and improves the performance of the deep network. DRCN [16] and DRRN [17] use a recursive approach and parameter sharing strategy to reduce parameters further but increase the depth and width of the network. Zhang et al. [18] proposed a residual dense network (RDN) with dense skip connections and residual structure that can capture more contextual information to reconstruct images.

Most of the above approaches are focused on improving performance by designing wider and deeper network. Still, as the network depth and width increase, the computational requirements and memory consumption also increase, making deep networks unsuitable for applications on mobile devices. Moreover, the deepening of the network causes the low-dimensional information of the image to fade away in the continuous nonlinear mapping, which is not conducive to the reconstruction of high-quality images. Therefore, Ahn et al. [19] proposed the lightweight cascading residual network CARN-M, which replaces the vanilla convolution with group convolution to speed up the network inference while reducing the number of parameters. Hui et al. [20] proposed an information distillation network (IDN), which improves the expressiveness of the network by combining the output relevant information with the redundant feature information obtained from distillation. However, these approaches reduce parameters at the cost of substantial performance and do not achieve a favorable trade-off. Then, Hui et al. improved the IDN by proposing the information multidistillation network (IMDN) [22]. IMDN designed an information multi-distillation block (IMDB) to progressively extract helpful information and aggregate two different features, achieving a good trade-off between network complexity and reconstruction quality. Nevertheless, although IMDN reduces the number of network parameters, it sacrifices part of the performance and cannot fully utilize the representational power of convolutional neural networks.

To further improve the performance of the lightweight super-resolution model, we elaborately design a lightweight image super-resolution network based on re-parameterization and self-calibrated convolution, named RepSCN. Due to the excessive amount of deep neural network parameters and the computational resources required, we follow the shallow network structure of IMDN. Considering that information multidistillation block (IMDB) in IMDN employs channel splitting operation to extract features, making features inconsistent in the number of channels before and after convolution, inconvenient to benefit from residual learning using identity connection, and brings inflexibility to the network structure design. To improve the inferential and representational power of the network, we designed a re-parameterization distillation block (RepDB) and a self-calibrated distillation block (SCDB) to replace the IMDB. In the shallow feature extraction stage, the re-parameterization convolution (RepConv) in RepDB can collect more useful information than the standard convolution without introducing extra cost in the inference phase. In the deep feature extraction stage, the self-calibrated block (SCB) with a more extensive convolutional receptive field works as the feature extraction module of SCDB, which can help the network to generate feature maps containing rich high-frequency details. It is worth mentioning that RepDB and SCDB do not introduce additional parameters. On the other hand, lightweight models with a small number of parameters limit the SR performance improvement. The contrast-aware attention (CCA) layer in IMDN only learns feature mappings from the channel dimension, which is inefficient. Therefore, we choose to introduce a lightweight coordinate attention mechanism (CAM) [22] at the end of RepDB and SCDB, which captures not only cross-channel but also direction-aware and position-sensitive information. It can be demonstrated through comparative and ablation experiments that the proposed network structure achieves high SR quality while maintaining a modest model size.

For this paper, the main contributions are as follows:

1. We, for the first time, introduce the idea of structural re-parameterization in the distillation network and propose a re-parameterization distillation block (RepDB) to speed up the inference of the model while further improving the performance of SR reconstruction.
2. We propose a self-calibrated distillation block (SCDB) with a self-calibrated block (SCB) to increase the receptive field of convolutional layers, which can generate features containing more contextual information without introducing additional parameters.
3. Based on RepDB and SCDB, we design a lightweight and efficient SR network (RepSCN), which can fuse multiscale features under different receptive fields to enhance feature representation. A coordinate attention mechanism (CAM) is also introduced to further improve performance. Numerous experiments have demonstrated that RepSCN achieves comparable SR performance with state-of-the-art models while using a modest number of parameters.

## 2. Related Work

### 2.1. Singe-Image Super-Resolution

Recently, deep learning models have dramatically advanced the development of single-image super-resolution (SISR) tasks. Dong et al. [12] first combined deep learning techniques with SISR and proposed a network (SRCNN) consisting of three convolutional layers to learn the mapping between HR images and LR images in an end-to-end manner. Compared with SRCNN, ESPCN [23] designed a subpixel convolution layer to upsample the feature maps to the target size only at the end part of the network, greatly reducing the computational and storage complexity of the model. VDSR [14] introduced residual learning to tackle the problem of difficulty in training deep networks, and SR performance has improved with the deepening of the network. Later, to reduce the number of network parameters, Kim et al. [16] proposed a novel recursive network DRCN that achieves good performance using a parameter sharing strategy. LapSRN [24] used a pyramid framework to gradually enlarge the size of the input image patch. Tai et al. [25] proposed a persistent memory network (MemNet), which merges previous feature information using skip connections and solves the long-term dependency problem of deep models. EDSR [15] removes the BN layer in residual blocks, based on which RDN [18] introduces the dense connections, which reduces the parameters and improves the performance compared to EDSR. RCAN [26] introduced the channel attention mechanism to form a new residual structure. SRFBN [27] proposes a feedback mechanism to improve the representational power of the network.

To better deploy the model on mobile devices, Ahn et al. [19] proposed CARN, which uses a recursive cascading mechanism to learn multilevel feature representations. IDN [20] effectively combines local long and short path features using group convolution. IMDN [27] proposes an information multiple-distillation block (IMDB) that extracts hierarchical features using channel split operation. Later, RFDN [28] improved IMDB with two parallel convolutional operations to separate the feature channels. FDIWN [29] proposed the Wide-residual Distillation Interaction Block (WDIB) to interact features with different scales. LBNet [30] integrates CNN and Transformer for building a more efficient model.

In perceptual-driven methods, Ledig et al. [31] proposed a generative adversarial network (GAN)-based model SRGAN with a new perceptual loss function defined. Then, ESRGAN [32] introduced a Residual-in-Residual Dense Block (RRDB) on the top of SRGAN to enhance the visual quality further. However, although GAN-based models can generate finer texture details, there is always the problem of geometric structure distortion in the recovered images.

### 2.2. Attention Mechanism

The attention mechanism is a mechanism for resource allocation, and in computer vision tasks, it is used to find correlations between data and then focus on certain important features. Hu et al. [33] proposed a squeeze-and-excitation network (SENet) that learns the degree of dependency of each channel and redistributes channel feature information according to the interdependence between channels. After that, considering that channel attention can effectively help the network to learn the high-frequency information of images in SR tasks, Zhang et al. [26] introduced the channel attention mechanism into the residual learning-based block and proposed the RCAN model. The Efficient Channel Attention (ECA) module [34] improves SENet by generating channel attention via fast 1D convolution and is suitable for application in lightweight networks. Moreover, combining channel and spatial attention is an important development in attention mechanisms. CBAM [35] inferred attention weights along both spatial and channel dimensions. SRRAM [36], on the other hand, proposed a residual attention module (RAM) based on CBAM that is more suitable for SR tasks. Recently, Wang et al. [37] proposed a balanced attention mechanism (BAM) for SISR, combining the structure of MaxPool for spatial attention and AvgPool for channel attention, which is lightweight and efficient. Due to the effectiveness of the attention model, our network introduces a coordinate attention mechanism [22] in the local feature aggregation part to further enhance the network performance.

## 3. Proposed Methods

### 3.1. Network Framework

The overall framework of the proposed network is illustrated in Figure 1, and our RepSCN consists of four parts: feature extraction module, nonlinear feature mapping module, feature fusion part, and reconstruction module.  Algorithm 1 formulates the network forward step. Taking **I**_*LR*_ and **I**_*SR*_ as the input and output of the network, respectively, the feature extraction module is composed of a convolutional layer with 56 channels and 3 × 3 kernel size, which can be expressed as follows:

(1) $$\begin{array}{c} F_{0}=f_{s}\left(I_{LR}\right), \end{array}$$

where *f*_*s*_(*·*) denotes the shallow feature extraction function. After that, the shallow feature **F**_0_ is fed to the nonlinear feature mapping module for extracting useful feature information, which consists of three re-parameterization distillation block (RepDB) and three self-calibrated distillation block (SCDB) stacked in a chain-like manner, as shown in the following equation:

(2) $$\begin{array}{c} F_{i}=f_{\text{Rep}DB}\left(F_{i-1}\right),\;i=1,\ldots ,n,\\ F_{j}=f_{SCDB}\left(F_{j-1}\right),\;j=n+1,\ldots ,n+m, \end{array}$$

where *f*_RepDB_(*·*) and *f*_SCDB_(*·*) denote the RepDB function and SCDB function, respectively. **F**_*i*−1_ and **F**_*i*_ represent the input and output features of the *i*-th RepDB, and similarly, **F**_*j*−1_ and **F**_*j*_ represent the input and output features of the (*j* − *n*)-th SCDB, respectively. All these intermediate features are aggregated together by a concatenation operation, and then a 1 × 1 and 3 × 3 convolutional layer is used to compress the feature channels and further refine the features. The feature fusion part can be formulated as follows:

(3) $$\begin{array}{c} F_{f}=f_{f}\left(\text{cat}\left(F_{1},\ldots ,F_{n},\ldots ,F_{m}\right)\right), \end{array}$$

where cat(*·*) stands for the concatenation operation of channel dimension and*f*_*f*_(*·*) is the 1 × 1 convolution and 3 × 3 convolution. Finally, the aggregated feature**F**_*f*_and shallow feature **F**_0_ are element-wise summed and upsampled to the target size by the upsampling reconstruction module as follows:

(4) $$\begin{array}{c} I_{SR}=f_{\text{rec}}\left(F_{f}+F_{0}\right), \end{array}$$

where *f*_rec_(*·*) denotes the reconstruction module, which upsamples the image using subpixel convolution to obtain the reconstructed SR image.

We denote the training set as {**I**_*HR*_^*t*^, **I**_*LR*_^*t*^}_*t*=1_^*T*^, which contains *T* iterations of all LR-HR image pairs. The loss function of our RepSCN can be described as

(5) $$\begin{array}{c} ℒ\left(\theta \right)=\frac{1}{T}\overset{T}{\underset{t=1}{\sum }}\left\|I_{HR}^{t}-f_{\text{RepSCN}}\left(I_{LR}^{t}\right)\right\|1, \end{array}$$

where *θ* represents all learnable parameters in the network and *f*_RepSCN_(*·*) is our RepSCN function. ||*·*||_1_ means the L1 norm.

### 3.2. Re-Parameterization Distillation Block

As shown in Figure 2, our re-parameterization distillation block (RepDB) consists of cascaded re-parameterization convolutions (RepConv), 1 × 1 convolution, and 3 × 3 convolution for reducing the number of feature channels and coordinate attention mechanism (CAM). The whole module utilizes residual connections to extract valuable features progressively.

In Figure 2, inspired by RFDN [28], the feature distillation operation is implemented by a 1 × 1 convolution that compresses the feature channels at a rate of 0.5, and the re-parameterization convolution is utilized to refine the features little by little. Given an input feature **F**_in_, the process of the *i*-th RepDB can be formulated as follows:

(6) $$\begin{array}{c} F_{\text{distill}\_1}^{i},F_{\text{refine}\_1}^{i}=D_{1}^{i}\left(F_{\text{in}}^{i}\right),R_{1}^{i}\left(F_{\text{in}}^{i}\right),\\ F_{\text{distill}\_2}^{i},F_{\text{refine}\_2}^{i}=D_{2}^{i}\left(F_{\text{refine}\_1}^{i}\right),R_{2}^{i}\left(F_{\text{refine}\_1}^{i}\right),\\ F_{\text{distill}\_3}^{i},F_{\text{refine}\_3}^{i}=D_{3}^{i}\left(F_{\text{refine}\_2}^{i}\right),R_{3}^{i}\left(F_{\text{refine}\_2}^{i}\right),\\ F_{\text{refine}\_4}^{i}=R_{4}^{i}\left(F_{\text{refine}\_3}^{i}\right), \end{array}$$

where **F**_distill_*j*_^*i*^ and **F**_refine_*j*_^*i*^ represent the *i*-th distilled feature and refined feature of the *j*-th RepDB, respectively. *R*_1_^*i*^,*R*_2_^*i*^,*R*_3_^*i*^ represent the three re-parameterization convolutional layers of the *i*-th RepDB, and *R*_4_^*i*^ is a 3 × 3 convolutional layer to decrease the number of channels of the refined features. *R*_*j*_^*i*^ represents the *j*-th 1 × 1 convolutional layer of the *i*-th RepDB. Then, the distilled features and the final refined feature are concatenated together and added to the input feature **F**_in_ to obtain the output feature **F**_out_ of the module. It can be expressed as follows:

(7) $$\begin{array}{c} F_{\text{out}}=f_{\text{CAM}}\left(f_{C}\left(\text{cat}\left(F_{{\text{distill}}_{1}}^{i},F_{{\text{distill}}_{2}}^{i},F_{{\text{distill}}_{3}}^{i},F_{{\text{refine}}_{4}}^{i}\right)\right)\right)+F_{\text{in}}, \end{array}$$

where cat(*·*) is a concatenation operation in channel dimensions and *f*_*C*_(*·*) denotes a 1 × 1 convolution used to compress feature channels to the same size as the input features. *f*_CAM_(*·*) is the coordinate attention mechanism.

Since the multibranch structure can lead to high-performance benefits for the network, inspired by RepVGG [38], we propose a re-parameterization convolution (RepConv) based on the RepVGG block but more applicable for SR tasks. Unlike the RepVGG block, as shown in Figure 2, RepConv removes the BN layer that is ineffective for the SR task. In the training phase, RepConv can be represented as *y* = *g*(*x*) + *f*(*x*) + *x*, where *g*(*x*) and *f*(*x*) correspond to 1 × 1 convolution and 3 × 3 convolution, respectively. Although we can obtain various receptive fields by employing different convolution kernels on different branches, the multibranch structure is slower during inference and has an increased memory occupation.

To address the above problem, we transform the trained multipath model into a single-path model in the inference phase. The specific procedure is shown in Figure 2. Given a re-parameterization convolution with the number of input channels and output channels both set to 2, the 1 × 1 convolution can be transformed into a 3 × 3 convolution by adding zero-padding. Setting the convolution kernel parameters of the current channel to 1 and the remaining channels to 0, the identity layer can also be transformed into the form of 1 × 1 convolution and further into 3 × 3 convolution. According to the principle of convolutional additivity, the convolutional layers in three branches are fused to form a new 3 × 3 convolution finally, and the bias of this 3 × 3 convolution is the sum of the bias of the previous 1 × 1 and 3 × 3 convolution. The experimental results show that the re-parameterization convolution can effectively improve the super-resolution reconstruction performance compared with the normal convolution.

### 3.3. Self-Calibrated Distillation Block

To recover more high-frequency details by using the low-frequency information of the image, we propose the self-calibrated distillation block (SCDB) to extract features in the deep network. As shown in Figure 3, the overall structure of the self-calibrated distillation block is the same as the re-parameterization distillation block, except that the re-parameterization convolution of the feature refinement part is replaced by a self-calibrated block, which can enlarge the receptive field of convolution and thus obtain richer contextual information, which helps to generate realistic HR images.

Inspired by SCNet [39], we improved the SCConv in SCNet by removing its BN layers and embedding a global residual connection to alleviate the pressure during training. The proposed self-calibrated block is shown in Figure 4, where the input features **X**_*n*−1_ are equally divided into **X**_*n*−1_′ and **X**_*n*−1_^″^ along the channel dimension by a 1 × 1 convolution. **X**_*n*−1_′ and **X**_*n*−1_^″^ are processed in two different branches, and the processed features are concatenated together and summed with **X**_*n*−1_to obtain the final output **X**_*n*_.

In the upper branch, we first perform an average pooling downsampling operation, a convolutional feature transformation operation, and a bilinear interpolation upsampling operation on the input features **X**_*n*−1_^'^, and then we sum it with the input feature to generate the spatial attention feature map. The spatial attention feature map is fused with the transformed **X**_*n*−1_′, and the output **X**_*n*_^'^ of this branch is obtained after a 3 × 3 convolution. The whole process can be expressed as follows:

(8) $$\begin{array}{c} X_{n}^{'}=f_{3}\left(f_{2}\left(X_{n-1}^{'}\right)*\sigma \left(f_{\text{Up}}\left(f_{1}\left(f_{\text{Down}}\left(X_{n-1}^{'}\right)\right)\right)+X_{n-1}^{'}\right)\right), \end{array}$$

where*f*_Up_(*·*) and*f*_Down_(*·*)denote the mean pooling upsampling operation and the bilinear interpolation upsampling operation, respectively. *f*_1_(*·*), *f*_2_(*·*), and *f*_3_(*·*) are 3 × 3 convolutions, and *σ*(*·*) is the sigmoid function.

In the lower branch, the input feature **X**_*n*−1_^″^ is fed into a 3 × 3 convolution layer to obtain the output **X**_*n*_^″^. **X**_*n*_^″^ is concatenated with the output **X**_*n*_′ of the upper branch and summed with the feature **X**_*n*−1_ containing a large amount of low-frequency information to generate the output **X**_*n*_ of the *n*-th self-calibrated block. This process can be formulated as follows:

(9) $$\begin{array}{c} X_{n}^{\prime \prime }=f_{4}\left(X_{n-1}^{\prime \prime }\right),\\ X_{n}=\text{cat}\left(X_{n}^{\prime \prime },X_{n}^{\prime }\right)+X_{n-1,} \end{array}$$

where *f*_4_(*·*) is the 3 × 3 convolution and cat(*·*) represents the concatenation operation along the channel dimensions.

### 3.4. Coordinate Attention Mechanism

The channel attention mechanism (e.g., SE Block in SENet [33]) can effectively improve the reconstruction performance but ignores the locational information, which is critical to capturing the spatial structure of the image in the SR task. CBAM [35] combines channel attention and spatial attention by feedforward propagation, which is likely to cause the loss of locational information. Therefore, to augment the feature representations of the network, we introduce the coordinate attention mechanism [22], which embeds locational information into channel attention and can learn long-range dependencies between spatial locations. It is also well adapted for application to lightweight SR models.

As shown in Figure 5, given an input **X** ∈ ℝ^56*∗H∗W*^, 56 is the number of feature channels of the input **X**, and *H*and *W*denote the height and width of the image, respectively. We utilize two spatially pooling kernels (*H*, 1) and (1, *W*) to encode each channel along the horizontal and vertical directions, respectively, and the output **Y** of the *c* -th channel at height *h* and width *w* can be formulated as follows:

(10) $$\begin{array}{c} Y_{c}^{h}\left(h\right)=\frac{1}{W}\underset{0\leq ,i\leq W}{\sum }X_{c}\left(h,i\right),\\ Y_{c}^{w}\left(w\right)=\frac{1}{H}\underset{0\leq j\leq H}{\sum }X_{c}\left(j,w\right). \end{array}$$

The above transformation obtains a pair of feature maps **Y**^*h*^ ∈ ℝ^56*∗H∗*1^ and **Y**^*w*^ ∈ ℝ^56*∗*1*∗W*^, and **Y**^*h*^ and**Y**^*w*^are concatenated together and then fed to a 1 × 1 convolution layer to generate the intermediate feature **F**. It can be described as follows:

(11) $$\begin{array}{c} F=\delta \left(f_{\text{conv}}\left(cat\left(Y^{h},Y^{w}\right)\right)\right), \end{array}$$

where cat(*·*) represents the concatenation operation along the spatial dimension, *f*_conv_(*·*) represents the 1 × 1 convolution, and *δ*(*·*) is the h-swish activation function. Then, we split **F**into **F**^*h*^and **F**^*w*^ along the spatial dimension and obtain the attention weights **Z**^*h*^ and **Z**^*w*^ by two 1 × 1 convolution transformations. The above process can be formulated as follows:

(12) $$\begin{array}{c} Z^{h}=\sigma \left(f_{h}\left(F^{h}\right)\right),\\ Z^{w}=\sigma \left(f_{w}\left(F^{w}\right)\right), \end{array}$$

where *σ*(*·*)is the sigmoid function. Finally, the input features**X**and attention weights **Z**^*h*^and **Z**^*w*^are multiplied to generate the output feature **Y**, which can be formulated as follows:

(13) $$\begin{array}{c} Y_{c}\left(i,j\right)=X_{c}\left(i,j\right)*Z_{c}^{h}\left(i\right)*Z_{c}^{w}\left(j\right). \end{array}$$

## 4. Experimental Results

### 4.1. Datasets and Evaluation Metrics

In our experiments, we use 800 high-quality RGB training images from the publicly available dataset DIV2K [40] as the training set to train our model. To test the performance of the model, we use four commonly used benchmark datasets: Set5 [41], Set14 [42], BSD100 [43], and Urban100 [44]. Set5, Set14, and BSD100 contain natural scene images, and Urban100 contains only urban scene images. In addition, we evaluated the SR results by calculating the widely used peak signal-to-noise ratio (PSNR) and the structural similarity index (SSIM) [45] on the Y channel of transformed YCrbr space.

### 4.2. Implementation Details

In the data preprocessing stage, the training set is augmented with data by horizontal and vertical flipping and 90°, 180°, and 270° rotations. Besides, we convert the HR images to the LR training images using a bicubic interpolation downsampling operation in MATLAB.

In the training stage, the input image patch size is 64 × 64. We optimize the model using ADAM algorithm with parameters set to *β*_1_ = 0.9, *β*_2_ = 0.999, and *ϵ*=10^−8^. The batch size is set as 32, and the initial learning rate is set to 5*e* − 4 and is reduced by half every 200 epochs for a total of 1000 epochs.

The ×2, ×3, and ×4 models are trained from scratch when training the final models. The entire network is implemented on the PyTorch framework with an NVIDIA RTX 3080 GPU.

### 4.3. Ablation Study

In this section, we will discuss the differences between our proposed method and IMDN [27]. As shown in Figure 6, we designed four blocks that each forms the body part of the network shown in Figure 1 in a stacked manner, based on which we conducted ablation experiments to validate the effectiveness of each of the proposed blocks. The structure of IMDB, the building block of IMDN, is shown in Figure 6(a). The channel splitting operation limits the number of channels before and after feature extraction, making it difficult to introduce identity connections. Therefore, we designed the feature distillation block (FDB) shown in Figure 6(b), which uses 1 × 1 convolution for channel reduction and is more flexible than IMDB.

Table 1 shows the results of the ablation experiments. From the first two rows of Table 1, we observe that FDB improves the performance compared to IMDB, and the PSNR value increases by 0.05 dB on the Urban100 dataset. In the second and third rows, the coordinate attention mechanism (CAM) achieves better experimental results than the contrast-aware channel attention layer (CCA Layer) with approximately the same number of parameters. By comparing the last four rows, we can see that both the re-parameterization convolution (RepConv) and the self-calibrated block (SCB) can bring significant performance benefits to the SR network after replacing the standard convolution, and the combination of the re-parameterization distillation block (RepDB) and the self-calibrated distillation block (SCDB) can maximize this benefit when used together. Thus, we choose 3RepDB + 3SCDB as the main structure of the proposed RepSCN. Comparing the first and last rows, we can observe that RepSCN outperforms IMDN on each data set with the same experimental settings, especially on the Urban100 dataset, where the PSNR value improves by 0.20db and the SSIM value improves by 0.0055.

### 4.4. Model Complexity Analysis

The number of model parameters is an important metric to evaluate the complexity of a lightweight network. To directly show that the proposed RepSCN method obtains better SR results with fewer parameters, we compared RepSCN with the following 13 lightweight networks on ×2 Urban100 dataset: SRCNN [12], FSRCNN [13], VDSR [14], DRCN [16], DRRN [17], LapSRN [24], MemNet [25], IDN [20], EDSR-baseline [15], SRMDNF [46], CARN [19], MADNet [47], and IMDN [27]. As shown in Figure 7, we can see that our RepSCN outperforms the other lightweight networks by a large margin while maintaining a modest model size.

The number of Mult-Adds is another important metric to measure the complexity of the SR model.  Figure 8 shows the effect of Mult-Adds against PSNR for RepSCN and mainstream lightweight networks on the Urban100 ×2 dataset. We can find that RepSCN achieves better reconstruction results with fewer Mult-Add operations than other lightweight networks.

### 4.5. Comparison with State-Of-The-Arts

To intuitively show the effectiveness and efficiency of the proposed RepSCN model, we compared our RepSCN with various lightweight SR methods, including SRCNN [12], FSRCNN [13], VDSR [14], DRCN [16], LapSRN [24], MemNet [25], IDN [20], EDSR-baseline [15], SRMDNF [46], CARN [19], MADNet [47], IMDN [27], MSICF [48], and MSWSR [49]. To make a fair comparison with the above methods, we train our models individually for the scaling factors of ×2, ×3, and ×4.

Table 2 shows the number of parameters and objective evaluation metrics values for different models on the four benchmark datasets. We can see that the experimental results of IMDN are better than those of other methods except RepSCN at the upscaling factor of 2×. However, when the scale factor is set to ×4, the experimental results of IMDN are not as well compared with CARN and EDSR because CARN and EDSR with deeper and wider network structures can learn more feature information on large-scale datasets. Our proposed RepSCN has the same depth as IMDN, but by merging RepDB with SCDB, we obtain a larger receptive field and significantly enhance the representational power of the network. As a result, RepSCN achieves the best reconstruction performance on all four benchmark datasets with different upsampling factors, especially on the Set14 and Urban100 datasets, where the average PSNR values improve by 0.05 dB and 0.15 dB compared to IMDN, and the average SSIM values improve by 0.0013 and 0.0034 compared to IMDN, respectively. In summary, our RepSCN achieves the best trade-off against other lightweight methods in terms of performance and parameters.

### 4.6. Qualitative Comparisons

Figure 9 shows the subjective visual effect on scale ×4 from the Urban100 dataset. As can be seen from images “Img044” and “Img085,” most of the compared methods suffer from severe blurring artifacts, in contrast to our RepSCN, which produces more accurate lines and reconstructs more high-frequency details. From the image “Img025,” we observe that other methods produce the wrong reconstruction of the image texture direction to some extent. RepSCN can recover clear and correct texture details and generate more realistic visual results.

## 5. Conclusion

In this work, we propose a lightweight convolutional neural network based on re-parameterization and self-calibrated convolution for SISR. Specifically, we design the re-parameterization distillation module (RepDB) and the self-calibrated distillation module (SCDB) as the building blocks of the SR model. RepDB and SCDB can aggregate local features from different stages to obtain a more powerful feature representation, and re-parameterization convolution (RepConv) and self-calibrated blocks (SCB) are used to extract features at a fine-grained level. Moreover, we introduce the coordinate attention mechanism (CAM) to obtain long-distance dependencies between different locations, which is beneficial to recover more high-frequency details. Numerous experiments show that our method can achieve comparable performance with state-of-the-art lightweight networks. Our RepSCN reconstructs high-quality images with a small number of parameters.

In the future, we will explore more efficient re-parameterization strategies and use a single-branch network structure to accelerate model inference, which allows our models to be embedded in edge devices. In addition, we will also apply our approach to other image processing fields such as hyperspectral remote sensing and medical imaging.

## Figures and Tables

**Figure 1:** Architecture of the proposed framework.

**Figure 2:** The left figure shows the architecture of our proposed reparameterization distillation block (RepDB). The right figure presents the reparameterization convolution (RepConv). Here, the number of input channels and the number of output channels both are set to 2, so a convolution layer has four matrices.

**Figure 3:** Architecture of our proposed self-calibrated distillation block (SCDB).

**Figure 4:** Architecture of our proposed self-calibrated block (SCB).

**Figure 5:** Architecture of coordinate attention module (CAM).

**Figure 6:** Structure diagrams of different building blocks used in the ablation study (a) IMDB, (b) FDB, (c) RepDB and (d) SCDB.

**Figure 7:** Trade-off between performance and number of parameters on Urban100 dataset with scale factor ×2.

**Figure 8:** PSNR performance versus Mult-Adds on Urban100 dataset with scale factor ×2.

**Figure 9:** Visual comparisons of RepSCN with other SR methods on Urban100 dataset with scale factor ×4.

**Algorithm 1:** RepSCN function.

**Table 1:** Ablation studies of the effects of IMDB, FDB, RepDB, and SCDB with ×4 scale factor on test sets.

Method	Scale	Params (K)	Set5 PSNR/SSIM	Set14 PSNR/SSIM	BSD100 PSNR/SSIM	Urban100 PSNR/SSIM
6IMDB	×4	715	32.15/0.8940	28.56/0.7808	27.54/0.7348	25.97/0.7826
6FDB + CCA	×4	737	32.16/0.8943	28.58/0.7814	27.55/0.7348	26.02/0.7831
6FDB + CAM	×4	742	32.17/0.8946	28.59/0.7816	27.55/0.7355	26.05/0.7842
6RepDB	×4	742	32.20/0.8948	**28.61**/0.7818	27.56/0.7356	26.09/0.7862
6SCDB	×4	801	**32.23**/0.8951	**28.61**/0.7819	27.57/0.7359	26.11/0.7863
3RepDB+3SCDB	×4	772	32.22/**0.8953**	**28.61**/**0.7820**	**27.58**/**0.7363**	**26.17**/**0.7881**

**Table 2:** Average PSNR (dB)/SSIM values with the scale factors ×2, ×3, and ×4 on Set5, Set14, BSD100, and Urban100. The best performance is highlighted in **red**, and the second-best performance is highlighted in *blue*.

Method	Scale	Params	Set5 PSNR/SSIM	Set14 PSNR/SSIM	BSD100 PSNR/SSIM	Urban100 PSNR/SSIM
SRCNN [12]	×2	8K	36.66/0.9542	32.45/0.9067	31.36/0.8879	29.50/0.8946
FSRCNN [13]	×2	13K	37.00/0.9558	32.63/0.9088	31.53/0.8920	29.88/0.9020
VDSR [14]	×2	666K	37.53/0.9587	33.03/0.9124	31.90/0.8960	30.76/0.9140
DRCN [16]	×2	1774K	37.63/0.9588	33.04/0.9118	31.85/0.8942	30.75/0.9133
LapSRN [24]	×2	251K	37.52/0.9591	32.99/0.9124	31.80/0.8952	30.41/0.9103
DRRN [17]	×2	298K	37.74/0.9591	33.23/0.9136	32.05/0.8973	31.23/0.9188
MemNet [25]	×2	678K	37.78/0.9597	33.28/0.9142	32.08/0.8978	31.31/0.9195
IDN [20]	×2	553K	37.83/0.9600	33.30/0.9148	32.08/0.8985	31.27/0.9196
EDSR-baseline [15]	×2	1370K	37.99/0.9604	33.57/0.9175	32.16/0.8994	31.98/0.9272
SRMDNF [46]	×2	1511K	37.79/0.9601	33.32/0.9159	32.05/0.8985	31.33/0.9204
CARN [19]	×2	1592K	37.76/0.9590	33.52/0.9166	32.09/0.8978	31.92/0.9256
IMDN [27]	×2	694K	*38.00/0.9605*	*33.63/0.9177*	*32.19/0.8996*	*32.17/0.9283*
MADNet [47]	×2	878K	37.94/0.9604	33.46/0.9167	32.10/0.8988	31.74/0.9246
MSICF [48]	×2	4292K	*37.89/0.9605*	33.41/0.9153	32.15/0.8992	31.47/0.9220
MSWSR [49]	×2	1228K	37.49/0.9583	33.23/0.9123	31.88/0.8929	31.14/0.9169
RepSCN(Ours)	×2	753K	**38.01/0.9606**	**33.70/0.9192**	**32.19/0.8999**	**32.36/0.9307**
SRCNN [12]	×3	8K	32.75/0.9090	29.30/0.8215	28.41/0.7863	26.24/0.7989
FSRCNN [13]	×3	13K	33.18/0.9140	29.37/0.8240	28.53/0.7910	26.43/0.8080
VDSR [14]	×3	666K	33.66/0.9213	29.77/0.8314	28.82/0.7976	27.14/0.8279
DRCN [16]	×3	1774K	33.82/0.9226	29.76/0.8311	28.80/0.7963	27.15/0.8276
LapSRN [24]	×3	502K	33.81/0.9220	29.79/0.8325	28.82/0.7980	27.07/0.8275
DRRN [17]	×3	298K	34.03/0.9244	29.96/0.8349	28.95/0.8004	27.53/0.8378
MemNet [25]	×3	678K	34.09/0.9248	30.00/0.8350	28.96/0.8001	27.56/0.8376
IDN [20]	×3	553K	34.11/0.9253	29.99/0.8354	28.95/0.8013	27.42/0.8359
EDSR-baseline [15]	×3	1555K	*34.37/0.9270*	*30.28/0.8417*	*29.09/0.8052*	*28.15/0.8527*
SRMDNF [46]	×3	1528K	34.12/0.9254	30.04/0.8382	28.97/0.8025	27.57/0.8398
CARN [19]	×3	1592K	34.29/0.9255	30.29/0.8407	*29.06/0.8034*	28.06/0.8493
IMDN [27]	×3	703K	*34.36/0.9270*	*30.32/0.8417*	**29.09/0.8046**	*28.17/0.8519*
MADNet [47]	×3	930K	34.26/0.9262	30.29/0.8410	29.04/0.8033	27.91/0.8464
MSICF [48]	×3	4292K	34.24/0.9266	30.09/0.8371	29.01/0.8024	27.69/0.8411
MSWSR [49]	×3	—	−/−	−/−	−/−	−/−
RepSCN(Ours)	×3	761K	**34.49/0.9277**	**30.38/0.8433**	**29.09/0.8054**	**28.30/0.8553**
SRCNN [12]	×4	8K	30.48/0.8628	27.50/0.7513	26.90/0.7101	24.52/0.7221
FSRCNN [13]	×4	13K	30.72/0.8660	27.61/0.7550	26.98/0.7150	24.62/0.7280
VDSR [14]	×4	666K	31.35/0.8838	28.01/0.7674	27.29/0.7251	25.18/0.7524
DRCN [16]	×4	1774K	31.53/0.8854	28.02/0.7670	27.23/0.7233	25.14/0.7510
LapSRN [24]	×4	502K	31.54/0.8852	28.09/0.7700	27.32/0.7275	25.21/0.7562
DRRN [17]	×4	298K	31.68/0.8888	28.21/0.7720	27.38/0.7284	25.44/0.7638
MemNet [25]	×4	678K	31.74/0.8893	28.26/0.7723	27.40/0.7281	25.50/0.7630
IDN [20]	×4	553K	31.82/0.8903	28.25/0.7730	27.41/0.7297	25.41/0.7632
EDSR-baseline [15]	×4	1518K	32.09/0.8938	*28.58/0.7813*	*27.57/0.7357*	*26.04/0.7849*
SRMDNF [46]	×4	1552K	31.96/0.8925	28.35/0.7787	27.49/0.7337	25.68/0.7731
CARN [19]	×4	1592K	32.13/0.8937	*28.60/0.7806*	**27.58/0.7349**	*26.07/0.7837*
IMDN [27]	×4	715K	*32.21/0.8948*	28.58/0.7811	27.56/0.7353	26.04/0.7838
MADNet [47]	×4	1002K	32.11/0.8939	28.52/0.7799	27.52/0.7340	25.89/0.7782
MSICF [48]	×4	4292K	31.91/0.8923	28.35/0.7751	27.46/0.7308	25.64/0.7692
MSWSR [49]	×4	1228K	32.01/0.8914	28.47/0.7776	27.48/0.7311	25.78/0.7744
RepSCN(Ours)	×4	772K	**32.22/0.8953**	**28.61/0.7820**	**27.58/0.7363**	**26.17/0.7881**

## Data Availability

The data supporting the findings of this study are included within the article.
